The article "Evaluation of Cardiac Space-Occupying Lesions by Myocardial Contrast Echocardiography and Transesophageal Echocardiography" was retracted in 2023. Reasons: suspected computer-generated content; unreliable results or conclusions; lack of ethics approval or compliance; missing or withdrawn patient consent.

# Evaluation of Cardiac Space-Occupying Lesions by Myocardial Contrast Echocardiography and Transesophageal Echocardiography

**DOI:** 10.1155/2022/2066033

**Published:** 2022-01-25

**Authors:** Mingming Ren, Lei Huang, Xiaoqiang Ye, Zhifeng Xv, Chun Ouyang, Zhen Han

**Affiliations:** Department of Cardiovascular Surgery, Peking University Shenzhen Hospital, Shenzhen 518036, Guangdong, China

## Abstract

Heart space-occupying lesions are a disease that occurs frequently in clinical setting, and therefore, it is important to diagnose and treat this type of pathologies properly. Angiographic echocardiography and transesophageal sonogram are widely used for clinical diagnosis. Their application provides a guarantee for the diagnosis of cardiac space-occupying lesions. In this paper, the application of cardiac contrast echocardiography and transesophageal echocardiography in cardiac space-occupying lesions was studied. Prediction of cardiac lesions can accurately determine the nature of cardiac occupancies and provide a basis for clinical diagnosis and management judgments. The results of pathological analysis and experimental comparison showed that myocardial contrast echocardiography can accurately distinguish tumor and thrombus and make contribution to patients taking appropriate medical measures. At the same time, it can compare conventional transthoracic echocardiography and transesophageal echocardiography. The results showed that TEE could clearly show the cardiac lesions. The experimental data of 76.9% confirmed cases showed that the diagnostic accuracy is greatly improved. TEE can also clearly show small thrombus that TTE cannot, in which 2DTEE can clearly show the boundary between the space-occupying and surrounding tissues, and whether there is a clear boundary between the space-occupying and surrounding tissues is an important distinguishing point of benign and malignant tumors. In addition, the TEE probe can also be used for large angle imaging and multiangle rotation, so as to determine the tumor boundary and the spatial position relationship between the tumor and the surrounding tissue. All in all, myocardial contrast echocardiography and transesophageal echocardiography have better clinical application effect on cardiac space-occupying lesions.

## 1. Introduction

Space-occupying lesions are a special term in medical imaging diagnosis. The results appear in X-ray, B-ultrasound, CT, and other examinations. It points to something that is not grown out of the original part of an organ [1]. This kind of extra growth can press on the previous organ and cause a movement of the original apparatus. Space-occupying lesions usually include malignant or benign tumors, parasites, stones, and hematoma but are not caused by their own disease. Space-occupying lesions are different from cancers. In clinical examinations, experienced doctors can analyze the patient's condition through symptoms.

Heart-occupying lesions (that is, the growth of excess in the heart area will compress the heart) are one of the heart diseases that seriously threatens the life of patients [2]. The reason for space occupancy will differ depending on its size, the position, and whether it causes the symptoms and signs of blood fluids. Clinically, primary heart tumors, metastases, cancer thrombi, tumors, thrombi, etc. are common preoccupational lesions, the most common of which are tumors, thrombi, and primary heart tumors. Examination is particularly important when determining the disease, so an accurate examination should be performed.

In the study of heart-occupying lesions, many experts and scholars have conducted intensive research. Dong et al. studied four patients with space-occupying cardiomyopathy using electronic focusing high-resolution two-dimensional echocardiography [3]. In two patients with high-intensity echo clusters at different depths on the epicardial surface, histology confirmed the diagnosis of lymphosarcoma, showing patchy, malignant infiltration of varying thickness. The remaining two patients have very different characteristics: the lesion appears to be inherent to the left posterior wall. A patient with arrhythmia and a small package of noncontractive masses was histologically confirmed as rhabdomyosarcoma. In the second patient, histology confirmed fibroids. In these two patients, the location of the lesion has been determined by angiography [4]. Alexandra used transesophageal echocardiography (TEE) to detect the left atrium, revealing the potential source of cardiac embolism in 12 patients (26%). All patients had clinical evidence of heart disease. TEE detected 32 patients (69%) with potential source of cardiac embolism; 7 (21%) of them had no clinical evidence of heart disease. It was concluded that TEE is a technology superior to TTE, which can be used to identify potential sources of embolized heart and should be recommended for early treatment and prevention of further stroke in patients with potential heart disease or unexplained cerebrovascular accidents [5]. Italy's Ren and other agents have demonstrated improved image quality and diagnostic confidence, and its practicality is now widely accepted [6]. One of the advantages of contrast echocardiography is that it can integrate the best imaging of LV function (by analyzing wall motion) and myocardial perfusion imaging. In clinical trials, using various contrast agent-specific methods, several contrast agents have been shown to provide excellent myocardial contrast effects. In two recent studies evaluating stress ischemia, perfusion imaging by contrast echocardiography can provide more information than conventional wall motion analysis. The technique of deriving quantitative information from contrast echocardiographic images is still mainly used in research, not in clinical settings. Conclusion. Contrast echocardiography can comprehensively assess left ventricular function and myocardial perfusion, has a high spatial and temporal resolution, and has the potential for quantification [7, 8]. Machine learning is the study of how computers can simulate or implement human learning behavior in order to acquire new knowledge or skills and reorganize existing knowledge structures to continuously improve their performance; joint learning is a method in which two events are repeated in close proximity to each other in time, eventually forming connections in the brain over time.

This article briefly introduces the damage of heart-occupying lesions to patients and the application of new medical technology, introduces the application of ultrasound technology in the medical field, and further introduces myocardial ultrasound contrast and transesophageal echocardiography technology, using practical research methods. The application of myocardial contrast echocardiography and transesophageal echocardiography in heart-occupying lesions is analyzed. The incomparable results indicated that the use of cardiomyogram echocardiography and transesophageal sonography can effectively improve the diagnosis of an occupied cardiac lesion in patients. The next surgical steps for patients had contributed a lot.

## 2. Proposed Method

### 2.1. Heart Occupying Lesions and the Application of Ultrasound Technology

Space-occupying lesions are one of the more common clinical diseases. With the population aging in China, the growing incidence of cardiovascular and the rising incidence of cardiac preoccupying lesions has caused significant concern among a number of physicians and scholars. Space-occupying lesions include benign, malignant tumors, thrombosis, hematoma, and abscesses [9, 10]. The pathological classification of tumors is diverse, and common benign tumors include myxoma, lipoma, hemangioma, and rhabdomyosarcoma [11]. Malignant tumors include primary and secondary malignant tumors; the former is the most common sarcoma, and the latter is secondary to other organ tumors; the most common primary lesions are lung cancer, breast cancer, lymphoma, and liver cancer. Nonneoplastic lesions are often accompanied by a history of basic heart disease or cardiac surgery. Patients with thrombosis usually suffer from valve disease, dilated cardiomyopathy, or coronary heart disease. Patients with cardiac hematoma usually have a recent history of interventional therapy. Benign tumors can usually be cured by surgical removal. Based on the pathological and disease characteristics, we use chemotherapy, radiotherapy, and photoresection to be able to treat malignant tumors. Depending on the extent of the disease and the length of the medical history, nonneoplastic lesions are treated with drugs or surgery. It can be seen that the treatment methods for different types of space-occupying lesions are different [12, 13]. Therefore, it is particularly important to clarify the nature of space-occupying lesions before treatment.

With the advancement of technology, ultrasound technology has been applied in the medical field [14]. Compared with other medical shaping methods, ultrasound medical imaging technology has many advantages. It has no radiation, and in most cases, ultrasound diagnosis is noninvasive and will not cause harm to patients or doctors [15]. Therefore, ultrasonic medical imaging is considered a safe imaging method and has become a routine inspection method. In addition, ultrasound imaging equipment is relatively cheap, and the cost of diagnosis is relatively low. In addition, ultrasound can also image soft tissues, displaying the visceral anatomy and actual activity in real time. Therefore, at present, echocardiography has been widely used in the diagnosis of cardiovascular diseases. The heart is an organ with very complicated structure and movement. It is difficult to describe it accurately with traditional two-dimensional ultrasound, so in recent years, a three-dimensional reconstruction system of ultrasound medical images has emerged, using a series of two-dimensional ultrasound images in three-dimensional space. The three-dimensional shape of the heart is reconstructed, so that the heart can be observed from any angle, and some postprocessing methods are used to achieve accurate measurement of the heart cavity volume and free heart wall to achieve the purpose of accurate diagnosis [16, 17]. Ultrasound imaging is a new type of noninvasive diagnostic clinical medicine developed in the late 1950s. By studying the application of the physical properties and imaging rationale of ultrasound, as well as the knowledge of the anatomical, physiological, and pathological properties of human tissues and anatomies of organs and the basic knowledge of clinical physics, we observed the sound and image performance of human tissues, organ morphology, and function changes and then analyzed and discussed the occurrence and development of diseases, so as to achieve the purpose of disease diagnosis and treatment [18]. Transthoracic echocardiography (thoracic echocardiography, TTE) is one of the main methods for diagnosing heart-occupying lesions. It can observe the hemodynamic changes caused by the size, shape, location, and occupation of the space-occupying space in real time, but regarding this technique, due to its limitations, its results are susceptible to interference from many factors, such as the patient's body type. Such images are of poor quality and are not clear enough to define the specific spatial location of the lesion. It is easy to cause missed diagnosis and misdiagnosis, taking huge risks. Because of this, more precise methods and instruments are needed to accurately determine the type of lesion [19, 20]. In this form, ultrasound contrast and transesophageal echocardiography came into being [21, 22]. As early as the late 1980s, transesophageal echocardiography (TEE) was clinically applied, but the technology at that time was immature and, at the same time, affected by other factors such as cost; this technology has not been widely applied. Compared with transthoracic echocardiography, the transesophageal method can obtain a better acoustic window, thereby obtaining a better quality image of the heart [23, 24]. In particular, the development of real-time transesophageal three-dimensional echocardiography (RT3D-TEE) can display the heart in real time and three-dimensionally, providing clinicians with richer and more accurate information. In recent years, ultrasound contrast technology has been maturely used in the diagnosis of liver, thyroid, breast, and other organ occupying lesions. It can display the tiny blood vessels and low-speed blood flow of the occupying lesions, which helps evaluate its properties; there are also research applications. Myocardial contrast-enhanced ultrasound (MCE) determines the nature of cardiac tumors and believes that the degree of MCE enhancement can help distinguish between benign and malignant tumors [25, 26]. Computers can find patterns of heart disease onset and predict and evaluate heart disease with the help of different machine learning methods.

### 2.2. Myocardial Contrast Echocardiography and Transesophageal Echocardiography

Myocardial echocardiography (MCE) is currently a commonly used method for detecting cardiac function. In recent years, with the use of acoustic contrast agents, to observe myocardial perfusion by performing an echocardiogram has been made possible. This is known as myocardial echocardiography. It is also known as echocardiography of the corpus cavernosa. During the MCE examination, a specific microbubble contrast agent needs to be injected into the blood vessel. The microbubbles in the contrast agent are encapsulated by a high molecular weight gas (nitrogen or fluorocarbon gas) in a phospholipid or albumin shell. They cannot penetrate the endothelial cell layer and have similar dynamics to human red blood cells in blood vessels. They can be ruptured under the action of ultrasound and observed and recorded by relevant ultrasound equipment. The operation of heart echocardiography is simple, the cost is low, and there is no radiation. It is easier to be accepted by the majority of patients, and it has been gradually applied in clinical practice. In fact, the development of ultrasound contrast agents has also experienced three stages of leaping development; so far, the third generation of contrast agents has appeared [27, 28]. The first generation of contrast agents was produced in the 1980s. Its predecessor was a saccharide microbubble contrast agent. This discovery can be said to be a milestone in contrast agents. Since then, the development of ultrasonic microbubble contrast agents has entered an era of rapid development. Subsequently, some researchers obtained the transpulmonary circulation contrast agent with a diameter smaller than erythrocytes by acoustic vibration, which was the first generation of ultrasonic microbubble contrast agent. It was the first left heart acoustic contrast agent approved by the US FDA. The first generation of ultrasound microbubble contrast agent is also the first pulmonary transcontrast agent approved by the Ministry of Health of China. The second generation ultrasound microbubble contrast agent is mainly encapsulated with fluorocarbon gas or other inert gas, and its physical stability is improved compared with the first generation contrast agent. In addition, there are two kinds of contrast agent shells that are polymer composites, containing nitrogen or perfluorobutane, which can be used for cardiac cavity or myocardial imaging, have completed three key clinical trials, and have not yet officially put on the market. The third-generation targeted ultrasound microbubble contrast agent is still in the experimental stage. Generally speaking, the third-generation contrast agent is an improved version of the second-generation ultrasound microbubble contrast agent [29]. At present, myocardial ultrasound contrast is mainly used in the following aspects: application one to better identify the endocardial boundary: myocardial ultrasound contrast can better identify the endocardial boundary through enhanced cardiac cavity visualization, assess the wall thickness, and provide more accurate assessment. The left ventricular ejection fraction is also more accurate in evaluating the motor function of the wall segment. Diagnosis of two coronary heart diseases and evaluation of its therapeutic effect and prognosis is applied. Diagnosis of triple myocardial infarction and its complications is applied. We applied the diagnosis and characteristics of occupying lesions of the four cavities. MCE can detect the density of blood vessels in the space-occupying lesions in the heart, so as to roughly assess its properties. Intracardiac thrombus is generally free of blood vessels. MCE shows no obvious contrast agent filling; benign tumors in the heart generally have fewer blood vessels. MCE shows less contrast agent filling; and there are more blood vessels in cardiac malignant tumors, and MCE shows more abundant contrast agents. Filling: application of five cardiomyopathy diagnoses. Regarding hypertrophic cardiomyopathy, especially apical hypertrophy, MCE is a very good noninvasive diagnosis. Diagnosis of six myocardial insufficiency is applied. MCE can clearly show the boundary of the endocardium, can better find and diagnose the left ventricular nondensified myocardial segment, and can also identify asymptomatic myocardial densification patients early.

While the conventional transthoracic echo cardiogram can determine most of the oncotic lesions and is by far the most widely used means of visualization of oncotic lesions, its restrictions are also very well established. In order to be able to accurately determine the heart occupying, the nature of the lesions has been gradually applied and popularized by transesophageal echocardiography. In principle, transesophageal echocardiography (TEE) refers to an ultrasound imaging method, in which an ultrasound probe is placed in the esophagus to detect changes in the morphological structure and function of the heart and blood vessels from the back of the heart and blood vessels [30]. Its scanning method has undergone changes in single plane, double plane, and multiplane scanning and can be displayed more clearly. At present, multiplanar TEE has been widely used in the diagnosis of various heart diseases and the monitoring of thoracotomy and interventional surgery. Transesophageal echocardiography (TEE) was first used in the clinical field in the 1980s. Compared with transthoracic echocardiography, the transesophageal method can obtain a better acoustic window and thus a better quality of the heart. Image. Using the method of rotating transesophageal ultrasound probe to obtain two-dimensional sequence images of the heart and reconstruct the left ventricle to evaluate its morphology and volume, a microcontroller similar to an endoscope was designed to obtain multiplanar transesophageal echocardiography. With a modification of the esophageal ultrasound probe to control its rotation through a process to obtain pyramidal ultrasound montanic volume data, this method is utilized to the advantage of TEE to have a high quality reconstruction being achieved. In this paper, we have evaluated the diagnostic aspects of the prediction method and found that MCE is effective in differentiating between tumors and thrombi and improves the accuracy of the diagnosis of occupying lesions.

## 3. Experiments

### 3.1. Study of Myocardial Contrast-Enhanced Ultrasound on Heart Occupying Lesions

#### 3.1.1. Research Object

At a hospital, a total of 50 patients, 28 being men and 22 being women, aged 25–85 years, diagnosed with preoccupation of the heart by transthoracic radiology, were selected for the study. Patients diagnosed with the presence of cardiac thrombus based on clinical data, etiology, and TTE presentation were excluded. Of the 50 patients, 10 had previous history of malignant tumors of other organs; 45 tumors were confirmed by pathology, 5 tumors had reduced volume after chemotherapy, and 4 had reduced volume after thrombolytic therapy. Fifty patients were divided into benign tumor group (25 cases), malignant tumor group (20 cases), and thrombosis group (5 cases) according to clinicopathology and clinical diagnosis. This experiment is based on two latitudes of tumor detection time and size to determine tumor category. In general, tumors that do not change significantly in size over time are classified as benign. This example uses the most simplified two-dimensional model to visualize the sample data and produce the following graph, where the horizontal axis is the mass size, and the vertical axis is the time of detection. Each point represents the size of the tumor and the time of onset for a different patient, and the tumor is judged to be benign or malignant based on its color.

#### 3.1.2. Research Instruments

Using the PhilipsiE33 ultrasound system, the patient was lying on the left side, connected to an electrocardiogram, and conventional ultrasound was used to observe the size, shape, position, internal echo, and adjacent conditions of the tumor, and to store the image. Sign the informed consent for ultrasound imaging. Select an appropriate section, so that the tumor is displayed on the same section as the ventricular septum or the left ventricular posterior wall, enable the MCE mode, the mechanical index is 0.10, the frequency is 2.5∼3.5 MHz, and slowly push the Novi contrast agent 2.5 through the left median elbow vein ml, speed 1.25 mL/min, postinjection of normal saline 5 mL to flush the injection channel, observe the tumor and normal myocardial enhancement, and store dynamic images. Instruct the patient to keep quiet and not move during the entire imaging process.

#### 3.1.3. Research Methods

MCE semiquantitative analysis: visual observation: the degree of contrast enhancement of space-occupying lesions is divided into (1) high enhancement: the enhancement intensity inside the space-occupying lesion is higher than the adjacent myocardial tissue; (2) enhancement: enhancement intensity of the space-occupying lesion is equal to that of the adjacent myocardial tissue; (3) low enhancement: the enhancement intensity of the occupying lesion is lower than that of the adjacent myocardial tissue; (4) no enhancement: no enhancement agent is filled inside the occupying lesion. Diagnose malignant tumors with high-enhanced space-occupying lesions, whole-area-enhanced space-occupying lesions as normal myocardial tissue, and overall low-enhanced space-occupying lesions with benign tumors, and the morphological rules remain unchanged. The positional lesions were diagnosed as dense thrombi, and the space-occupying lesions that were significantly lobed after the angiography and had no internal enhancement were diagnosed as fresh thrombus with loose texture. The quantitative index of MCE uses the QLAB10.8 software computer region of interest ROI technology to select the region of interest and dynamically track it to obtain the contrast intensity-time curve of the heart-occupying lesion and the adjacent normal myocardium, and according to the formula *y* (*t*) = *A* (1 − *e* − *Bt*) + C line perfusion curve fitting, record the peak intensity *A* value of the space-occupying lesion and the adjacent myocardium (reflecting the blood volume of the area of interest), and record it as *A*1 and *A*2, respectively, and calculate *A*1/*A*2 ratio; the ratio is greater than 1 diagnosed as malignant tumor, the ratio is diagnosed as benign tumor or thrombosis in the range of (0,1), and the ratio is equal to 0 diagnosed as thrombosis. Use SPSS18.0 professional statistical software analysis. MCE semiquantitative index results are adopted. The absolute value indicates that the chi-square test is used to compare the semiquantitative indexes of MCE between benign and malignant heart tumor groups; the results of the quantitative indexes of MCE are described by *x* ± *s*, and the independent sample *t*-test is used to compare the quantitative indexes of MCE between benign and malignant heart tumor groups; *P* < 0.05 means that the difference was statistically significant.

### 3.2. Transesophageal Echocardiography Study of Heart Occupying Lesions

#### 3.2.1. Research Object

52 patients were selected for TEE examination in a hospital, 22 males and 30 females, aged 20–60 years. Of the 52 cases, 8 had no obvious symptoms, and the physical examination found that the heart occupied, and the remaining 44 had obvious symptoms and signs (including varying degrees of palpitations, shortness of breath, chest tightness, heart murmur, and 10 of them with brain Infarction). Examination found that the heart occupied space. Ten of 52 patients occupy a history of malignant tumor. An occupying lesion is a general term for a group of conditions, in which the body's tissues occupy a certain spatial position. The majority of occupying heart lesions are caused by heart disease, but some are also caused by bruising inside the heart or by cysts.

#### 3.2.2. Research Instruments

Ultrasonic examination uses Philips iE33 colour ultra-Doppler ultrasound diagnostic instrument, equipped with C5-1 transthoracic probe and X7-2t three-dimensional transesophageal real-time probe. Transesophageal real-time 3D has a real-time three-dimensional display mode (Live-3D) and ECG-gated three-dimensional full-volume display mode (3DFullVolume).

#### 3.2.3. Research Method-Comparative Analysis of Conventional Transthoracic Echocardiography and Transesophageal Echocardiography

TTE examination method: first, let the patient take the supine position, with the left ventricular long-axis view, left ventricular short-axis view, left ventricular apex four-chamber view, etc. as the standard part of cardiac ultrasound scanning. To measure the size of each cardiac chamber regularly and to attentiveness to the specific characteristics of the defect and its association with the surviving tissues. TEE examination method: before the examination, it is necessary to make sure that the patient has no contraindications, the consent form has been signed, and the examination room is equipped with the necessary first aid equipment. Instruct patients to fast for more than 16 hours, take the left position, connect the ECG; use X7-2t probe, 2DTEE multi-angle scanning observation, measure relevant indicators and store images and data; then, use RT3DTEE imaging; first use real-time 3D mode display, observe the position, shape, and size of the cardiac cycle, and then switch to 3DFullVolume (maximum fan angle width 104., thickness 101.) mode, adjust the fan angle and thickness, wide-angle display space, and surrounding structure, and continuously store 4∼7. During the cardiac cycle, rotate and cut the stored 3DFullVolume image, observe carefully, clearly show the lesion, and measure its maximum footprint. Using SPSS18.0 software analysis, the maximum meridian of the space-occupying lesion is represented by *z* ± *s*. Use the ￡ test to compare the size of the heart-occupying lesions measured by various methods with the size of pathological specimens, and the size of the heart-occupying lesions measured by various methods, and compare the size correlation using the pathological specimens Pearson method. *P* < 0.05 indicates that the difference is statistically significant.

## 4. Discussion

### 4.1. Analysis of Myocardial Ultrasound Contrast Results

#### 4.1.1. Pathological Results

Of the 50 heart-occupying cases, 25 cases were (25/50, 50%) in the benign tumor group, including 15 cases of myxoma, 3 cases of lipoma and hemangioma, 2 cases of fibroids, and 2 cases of intracardiac leiomyoma, and 25 benign tumors were confirmed by surgery: 20 cases of malignant tumors (20/50, 40%), including 8 cases of lung cancer heart metastasis, 3 cases of malignant thymoma heart metastasis, and 3 cases of liver cancer heart metastasis and lymphoma and pericardial osteosarcoma. Pericardial angiosarcoma and neuroectodermal malignant tumors each had a heart metastasis; 20 cases of malignant tumors were confirmed by surgery in 10 cases (3 cases of malignant thymoma, liver cancer heart metastasis, lung cancer heart metastasis 2 cases, pericardial osteosarcoma, pericardial angiosarcoma 1 in each case of lymphoma), 7 of the remaining 10 unoperated patients had shrinkage after chemotherapy (all lung cancer metastases), and 3 were confirmed by biopsy under CT biopsy (2 cases were neuroectodermal malignant tumors with heart metastasis, 1 (Case of lymphoma); 5 cases (5/50, 10%) in the thrombus group, based on medical history (respectively, chronic renal failure with central venous catheterization, 1 year after pulmonary valve stenosis, right atrial tumor (1 year after surgery and 5 years of palpitations) and TTE could not confirm the diagnosis of thrombosis, and they were included in this study, the volume after thrombolytic therapy is small, and final clinical diagnosis of cardiac thrombosis is applied.

#### 4.1.2. Analysis of Semiquantitative Indicators of Cardiac Space-Occupying MCE

See Table 1 for semiquantitative indicators of cardiac space-occupying MCE.

According to Table 1, in 25 cases of benign tumor group, 18 cases of tumor edge smoothing (18/25, 72%), 7 cases of tumor edge smoothing (7/25, 28%), of which 6 cases were myxoma intracardiac leiomyomatosis; 20 of 25 benign tumors showed low enhancement (20/25, 80%), 5 tumors showed high enhancement (5/25, 20%), and 3 were hemangiomas and 2 cases of lipoma; 17 of 25 cases of benign tumors showed uniform enhancement (17/25, 68%), 8 cases of tumors showed uneven enhancement (8/25, 32%), of which 3 cases were myxoma. There were 1 case of lipoma, 2 cases of hemangioma, and 1 case of intracardiac leiomyomatosis. In the 20 cases of malignant tumor group, 20 cases had uneven tumor edges (20/20, 100%); 20 cases had uneven enhancement (20/20, 100%); 14 of 20 malignant tumors showed high enhancement (14/20,70%), and 6 cases showed low enhancement, including 2 cases of lung cancer heart metastases, 2 cases of liver cancer heart metastases, and 2 cases of heart lymphoma. Of the thrombotic group, MCE displayed no enhancement in 5 cases. The semiquantitative results of MCE in the benign and malignant tumor groups were of statistical significance (*P* < 0.05). The results of MCE semiquantitative indicators of various tumors are shown in Table 2.

According to Table 2, 18 cases of myxoma in the benign tumor group showed low enhancement (18/18, 100%) after imaging, 6 cases showed uneven enhancement (6/18, 33.3%), and 8 cases had uneven edges. (8/18, 44.4%), and these 18 cases of myxoma showed typical changes; that is, they were all located in the atrium, the tumor pedicle was located in the oval fossa or the free wall of the atrium and lobulated, and the degree of activity was greater (14 can travel between the atrioventricular, 4 cases fluttered in the atrium with the cardiac cycle), combined with its MCE enhancement degree was diagnosed as a benign tumor with low blood supply; intraoperative and pathological findings showed 8 cases of myxoma tumors with uneven edges after angiography. It is lobulated, and thrombosis can be seen on the surface. Six cases showed unevenly enhanced tumor volume after angiography (4.3 mm × 4.9 mm∼4.2 mm × 6.9 mm), with brown or brown-red areas of visible calcification, fibrosis, and cystic changes. The posterior edges of 3 cases of lipoma MCE were smooth, but the degree of enhancement and the uniformity of the enhancement were different. During the operation, the tumor with uneven enhancement was larger in volume (5.2 cm × 5.6 cm), and old bleeding was seen inside.

#### 4.1.3. Analysis of Quantitative Indexes of Cardiac Tumor MCE

The quantitative index of cardiac tumor MCE is shown in Figure 1.

As can be seen from Figure 1, the curve obtained by the MCE quantitative analysis software shows that, in the malignant tumor group, 15 tumors in 20 cases had higher TIC than the surrounding myocardium, 5 tumors had lower TIC than the surrounding myocardium (2 cases of lung cancer metastasis, 2 cases of liver cancer heart metastasis Lymphoma), in 20 cases of benign tumor group, and 20 tumors had lower TIC than peripheral myocardium, 5 tumors had higher TIC than peripheral myocardium (3 hemangiomas, 2 lipomas), which was consistent with the semi-quantitative MCE enhancement index. Compared with tumor A/myocardial A and curve slope, the malignant tumor group was higher than the benign tumor group, and the differences were statistically significant; compared with the peak time (TTP), the malignant tumor group was lower than the benign tumor group, but the difference was not statistically significant.

Through the above analysis, the tumor and thrombus can be identified by MCE, and the thrombus MCE shows no enhancement; semiquantitative and quantitative indicators help judge the blood supply status of cardiac tumors: most benign tumors are of low enhancement, and there are also small ones in malignant tumors. Some have low enhancement; unevenly enhanced MCE and uneven edges have high diagnostic value for the diagnosis of malignant tumors; but for typical myxoma, the diagnostic value of conventional echocardiography is higher than MCE; for some tumors (this Lipoma, heart metastases of lung cancer, and lymphoma in the study), the same pathological type shows different degrees of enhancement, so more cases need to be collected for discussion. Secondly, MCE is different from the ultrasound contrast of liver, breast, thyroid, and other organs. First, MCE takes intravenous drip, which is different from intravenous bolus injection, so the heart develops longer, and the quantitative index results are different from other organs; second, the heart is a pulsating organ, which brings difficulties to MCE quantitative analysis. Software analysis will be affected by heart beats, especially tumors with long tumor pedicles. The operation of software analysis is more complicated; third, the requirements for the cut surface are more than others. Visceral ultrasonography is high, and MCE requires that the lesion is located at the same depth as normal tissue, so the operator is required to be proficient in each section of TTE, both to select a section to display the lesion and normal tissue at the same depth, but the depth cannot be too large; otherwise, the contrast of the effect is not good, and at the same time, it is necessary to avoid adverse factors such as rib sound windows.

### 4.2. Transesophageal Echocardiography Results Analysis

#### 4.2.1. Pathological Results

Pathological analysis is shown in Figure 2.

According to Figure 2, 30 of 52 cases of benign tumors (8 cases of hemangioma, 18 cases of myxoma, 2 cases of lipoma and 2 cases of fibroma) accounted for 57.7%, and all 30 cases were confirmed by surgery; cases accounting for 19.3%, of which 8 cases were confirmed by surgery, 6 cases of thrombosis accounting for 11.5%, significantly reduced after diagnosis by TEE and anticoagulation; 4 cases of thickened boundary ridge, accounting for 7.7%, diagnosed by TEE; two cases of hematoma, accounting for 3.8%, were confirmed by surgery. It is clear from this data that a large proportion of tumour cases are benign and can be diagnosed and treated with the aid of modern medical procedures.

#### 4.2.2. Results of Conventional Transthoracic Echocardiography and Transesophageal Echocardiography

An example of transesophageal echocardiography is shown in Figure 3.

The results of conventional transthoracic echocardiography and transesophageal echocardiography are shown in Figure 4.

It can be seen that Figure 4 compares the three sets of data in total, which are confirmed cases of 52 patients under the analysis of 2DTTE and TEE technology and cases of benign tumors and misdiagnosis. From the data comparison, we can see that the type of heart-occupying lesions in the 52 patients participating in the study was 20 cases diagnosed by 2DTTE, and the diagnosis rate was 38.5%. 40 cases were diagnosed by TEE, and the diagnosis rate was up to 76.9%. Under 2DTTE imaging, there were 30 cases of benign tumors, 12 cases were definitely diagnosed by 2DTTE, and 2 cases were misdiagnosed, while, under TEE imaging, 30 cases of benign tumors were diagnosed without misdiagnosis. It can be seen from the above that 2DTTE is subject to many restrictions in actual use, and it is easy to be interfered by internal and external factors to cause error in results, which may cause misdiagnosis and missed diagnosis. The diagnosis rate of TEE technology is much higher than 2DTTE.

Figure 5 is a comparison of three kinds of 2DTTE, 2DTEE, and RT3DTEE ultrasound methods to estimate the heart size and surgical specimens.

According to Figure 5, with the comparison of the size of the heart occupied by 2DTTE, 2DTEE, and RT3DTEE and the size of the surgical specimen, the difference is greater than the statistical value of 0.05, so there is no statistical significance. Based on the above research, we can draw the following conclusions: first, TEE technology can clearly show heart disease changes, greatly improving the accuracy of diagnosis, which is undoubtedly a huge boon for patients, greatly reducing the risk of misdiagnosis and missed diagnosis. As far as the research in this article is concerned, in 52 cases of experimental data, the diagnosis rate under 2DTTE imaging reached only 38.5%, less than half, while, under TEE technology, 40 cases were diagnosed, and the diagnosis rate was 76.9%, an increase of 100% compared with 2DTTE. The second is that the TEE technology can display the fine structure of the lesion more clearly, helping the surgeon make a more accurate diagnosis. For the present case, TEE may reveal tumor peduncles in 20 fibroid and 2 papillary elastic cases in this subset of vasculature. The third TEE imaging can clearly show the boundary between the occupying lesion and the surrounding tissue. In summary, TEE can not only improve the diagnosis rate, because of its clear image, but also help surgeons obtain more preoperative information, which helps make surgical plans.

## 5. Conclusions

It has to be said that heart occupation is one of the heart diseases that seriously threatens the lives of patients, and it will cause huge interference to patients and their families. The placeholder will show different symptoms and signs due to its own characteristics. Clinically, primary heart tumors, metastases, cancer thrombi, neoplasms, thrombi, etc. are all common heart-occupying lesions.

An investigation based on thermography echocardiography and transesophageal echocardiography in the clinical of occupant cardiac lesions is presented in this article. Cardiac echocardiography is simple to perform, is of low cost, and is radiation free. It is more acceptable to most patients and is gradually being used in clinical practice, but it is not possible to accurately determine the nature of the occupying cardiac lesion and to make the most accurate diagnostic modality. Using it, myocardial echocardiography and transesophageal echocardiography were in fact found to make an outstanding contribution to the diagnosis of occupying cardiac lesions.

Through the application study of myocardial contrast echocardiography and transesophageal echocardiography in the clinical practice of cardiac space-occupying lesions, the following conclusions are drawn: (1) MCE can effectively distinguish tumors from thrombus and thrombus and improve the accuracy of diagnosis of space-occupying lesions. (2) TEE can clearly show the change of heart disease. The experimental data confirmed 76.9% of the cases, and the diagnosis accuracy rate is greatly improved compared with 2D TTE (the diagnosis rate is only 38.5%). (3) TEE can also clearly display small blood clots, tumor pedicles, and other details and the boundary with the surrounding tissue, which is helpful to form a more accurate judgment. In summary, the application of myocardial contrast echocardiography and transesophageal echocardiography in the clinical practice of heart-occupying lesions is conducive to more comprehensive observation and evaluation of the diagnostic accuracy of heart-occupying lesions.

## Figures and Tables

**Figure 1:** Comparison of quantitative indexes of benign and malignant tumor group.

**Figure 2:** Transesophageal echocardiography results.

**Figure 3:** Example of transesophageal echocardiography.

**Figure 4:** Comparison of conventional transthoracic echocardiography and transesophageal echocardiography.

**Figure 5:** Comparison of the measured heart footprint with the size of the surgical specimen.

**Table 1:** Comparison of semiquantitative indexes in benign and malignant tumor group of heart.

Pathological diagnosis	Quantity	Is the far edge smooth after angiography		Whether the enhancement is even		Strengthen	
		Yes	No	Yes	No	Low	High
Malignant	20	0	20	0	20	6	14
Benign	25	18	7	17	8	20	5
*X* ^2^		19.2		19.2		11.8	
*P*		0		0		0	

**Table 2:** MCE semiquantitative indexes of different pathological types of cardiac tumors.

Pathological type	Quantity	Is the far edge smooth after angiography		Whether the enhancement is even		Strengthen	
		Yes	No	Yes	No	Low	High
Myxoma	18	10	8	12	6	18	0
Lipoma	3	3	0	2	1	2	1

## Data Availability

This article does not cover data research. No data were used to support this study.
